The article "Frequency of Acquired Renal Cystic Disease in Patients on Long-Term Hemodialysis and Associated Renal Cell Carcinoma" was published in 2022. Journal: Cureus.

# Frequency of Acquired Renal Cystic Disease in Patients on Long-Term Hemodialysis and Associated Renal Cell Carcinoma

**DOI:** 10.7759/cureus.24547

**Published:** 2022-04-28

**Authors:** Furqan Ali, Jibran Bin Aziz, Shahzaib Saleem, Sania Ishtiaq Khan, Saadat Khan, Sanam I Khan

**Affiliations:** 1 Dialysis, Diaverum Saudi Arabia, Al Namas, SAU; 2 Nephrology, University Hospital Limerick, Limerick, IRL; 3 Internal Medicine, Dr. Mohamad Amine Zbeib Polyclinic, Doha, QAT; 4 Paediatrics, University Hospital Limerick, Limerick, IRL; 5 Emergency Department, University Hospital Limerick, Limerick, IRL

**Keywords:** renal cell carcinoma (rcc), end stage renal disease (esrd), chronic renal failure, acquired cystic renal disease (acrd), hemodialysis

## Abstract

Background

Acquired cystic renal disease is one of the complications of end-stage renal disease (ESRD) patients on dialysis. We aimed to define the prevalence of acquired cystic renal disease in a dialysis center in a tertiary care setup in Pakistan.

Materials and methods

We conducted a cross-sectional study of 246 patients with ESRD from October 1, 2017, to March 30, 2018. We collected patient demographic data, comorbidities, duration (years), frequency (sessions/week), length of each dialysis session (hours), ultrasound findings, cystic renal disease occurrence, and associated complications for analysis.

Results

Our patient population consisted of 115 women (46.7%) and 131 men (53.3%) and had a mean age of 55.9 ± 15.1 years. Thirty-seven patients were on dialysis for one year, 78 (31.7%) for two years, and 131 (53.3%) for three or more years, as its more common with increasing duration. The mean dialysis duration was 2.3 ± 0.7 years. Of 246 patients, 49 (19.9%) had acquired cystic renal disease.

Conclusions

Given improved health care facilities, an increasing number of patients have a good survival on dialysis and develop long-term complications associated with end-stage renal disease, such as acquired cystic renal disease. Because the acquired renal cystic disease is associated with renal cell carcinoma, physicians should evaluate dialysis patients for renal cell carcinoma, especially after three to five years of dialysis.

## Introduction

Pakistan's annual incidence of end-stage renal disease (ESRD) is estimated to be approximately 100 cases per million people [1]. Patients with ESRD experience several acute and chronic complications, including acquired cystic renal disease (ACRD). ACRD refers to the bilateral development of renal cysts in patients with ESRD caused by a primary non-cystic renal disorder [2]. The physical environment of chronic uremia in ESRD patients might facilitate cell division and inhibit apoptosis, leading to cyst formation and ACRD [3]. ACRD has been associated with a greater duration of dialysis; thus, in recent years, the incidence of ACRD has increased due to the longer survival of patients on dialysis [4]. ACRD is not associated with pain, unlike autosomal dominant polycystic kidney disease (ADPKD), but it is associated with a greater risk of cancer [5]. ACRD-associated renal cell carcinoma (RCC) is the most common tumor subtype in ESRD patients. This is especially concerning because the ESRD population has an up to 50 times greater risk of developing RCC than the healthy population [6]. Screening and early detection of dialysis patients every three years with computed tomography (CT) or ultrasound to detect ACRD can increase the life expectancy of patients with ESRD by one-and-a-half-years-a strategy that may be considered helpful in younger and healthier patients with fewer comorbidities than older patients [4]. The prevalence of ACRD increases with the duration of dialysis; approximately 90% of patients on dialysis for more than nine years have ACRD, 40% to 60% of patients on dialysis for more than five years have ACRD, and 20% of patients on dialysis for one to three years have ACRD [2]. No patients on dialysis for less than one year developed ACRD in the Pakistani population [7]; however, the sample size of that study was small, and most patients did not use dialysis for more than one year. There was no clinical or sonological evidence of RCC in these patients, and the prevalence of ACRD was 20.8% (18.9% in men and 22.6% in women). However, there is minimal data available from Pakistan regarding the prevalence of ACRD in patients on dialysis for more than one year. Therefore, we conducted this study to assess the current disease burden of ACRD in hemodialysis patients in the nephrology department of Shifa International Hospital in Islamabad.

The article "Frequency of Acquired Renal Cystic Disease in Patients on Long-Term Hemodialysis and Associated Renal Cell Carcinoma" was published in 2022. Journal: Cureus.

## Materials and methods

We conducted a cross-sectional study of patients treated at the dialysis unit of the Department of Nephrology, Shifa International Hospital in Islamabad, from October 1, 2017, to March 30, 2018. The study included men and women aged 18 to 70 years diagnosed with ESRD and receiving dialysis for longer than one year. We excluded any patients with known diagnosis of ADPKD, multiple cystic diseases, and previous ultrasound demonstrating cystic disease before the onset of dialysis from their available imaging studies. Furthermore, no patient had genetic testing for diagnosis. This study was approved by the Institutional Review Board (IRB) and Ethics Committee (EC) of Shifa International Hospital with approval number IRB# 645-093-2016. All participants provided written informed consent prior to data collection.

We collected detailed history, including age, sex, frequency and duration of dialysis, and length of each dialysis session. Patients underwent an ultrasonography examination of their kidneys, ureters, and bladders. We then assigned patients into three groups according to dialysis duration of one year, two years, or three or more years. We then noted the presence or absence of ACRD in each group. We used IBM Corp. Released 2019. IBM SPSS Statistics for Windows, Version 26.0. Armonk, NY: IBM Corp to analyze our results, and p<.001 was considered statistically significant.

## Results

The study population consisted of 246 participants with a mean age of 55.9 ± 15.1 years (range, 18 to 85 years). Over half the population were men (n=131, 53.3%), and 115 were women (46.7%). The patients underwent an ultrasound of their kidneys. Thirty-seven patients (15%) received dialysis for one year, 78 (31.7%) received dialysis for two years, and 131 (53.3%) received dialysis for three or more years. The mean duration of dialysis treatment was 2.3 ± 0.7 years at the time of ultrasound. Two hundred twenty-three patients (90.7%) received dialysis twice per week, and 23 patients (9.3%) received dialysis three cycles per week (Table 1).

**Table 1:** Study population demographic data

Demographic data	Frequency (%)
Sex	
Male	131 (53.3%)
Female	115 (46.7%)
Hemodialysis (Duration)	
1 year	37 (15.0%)
2 years	78 (31.7%)
≥3 years	131 (53. 3%)
Hemodialysis sessions/week	
2/Week	223 (90.7%)
3/Week	23 (9.3%)

Of 246 patients, 49 (19.9%) had ultrasonographic evidence of ACRD, and one patient (0.004 %) had RCC (Table 2). Only one patient had ACRD in the one-year dialysis group, and one patient had ACRD in the two-year dialysis group. Among the patients receiving dialysis for three or more years, 47 patients had ACRD (p<.001).

**Table 2:** Incidence of ACRD ACRD: acquired cystic renal disease.

	Yes	No	P-Value
ACRD Present, n (%)	49 (19.9%)	197 (80.1%)	
Presence of ACRD years of dialysis			
1 year	1 (0.020%)	36 (0.18%)	0.001 (for more than 3 years group)
2 years	1 (0.020%)	77 (39%)	
≥3 years	47 (96%)	84 (42.6%)	
Presence of ACRD by age in years			
˂20 years	2 (4.08%)	8 (4%)	0.511 (between age groups)
21-40years	3 (6.1%)	25 (12.6%)	
41-60 years	18 (36.7%)	83 (42%)	
61-80 years	25 (12.6%)	76 (38.5%)	
≥80 years	1 (2.04)	5 (2.5%)	

Among the 49 patients with ACRD, 32 (65.4%) were men, and 17 (34.6%) were women (p=0.059). ACRD was present in 39 patients receiving twice-weekly dialysis and 10 patients receiving thrice-weekly dialysis (p=0.003). Among those with ACRD, 14 had kidneys smaller than 7 cm, 30 patients had a kidney size of 7 cm to 9 cm, and five had a kidney measuring 10 cm to 12 cm (Table 3). We stratified patients by age and found that ACRD was present in two patients younger than 20 years, three patients aged 21 to 40 years, 18 patients aged 41 to 60 years, 25 patients aged 61 to 80 years, and one patient older than 80 years (Table 2).

The article "Frequency of Acquired Renal Cystic Disease in Patients on Long-Term Hemodialysis and Associated Renal Cell Carcinoma" was published in 2022. Journal: Cureus.

**Table 3:** ACRD presence by sex, dialysis frequency, and kidney size ACRD: acquired cystic renal disease.

ACRD by sex	Yes	No	P-Value
Male	32	99	0.059
Female	17	98	
ACRD by dialysis frequency			
Dialysis twice per week	39	184	0.003
Dialysis three times per week	10	13	
ACRD by kidney size			
10-12 cm	5	45	0.051 (Between groups)
7-9 cm	30	119	
˂7 cm	14	33	

## Discussion

To the best of our knowledge, this study represents the most extensive study to assess the presence of ACRD in a Pakistani population. ACRD was first described by Dunnil et al. in 1977 [8]. The condition is characterized by three or more cysts per kidney in a patient on dialysis without a hereditary cause of cystic diseases such as autosomal dominant polycystic kidney disease or tuberous sclerosis. Within the first three years of dialysis, approximately 10% to 20% of patients develop ACRD. By five years of dialysis, 40% to 60% of patients have ACRD, and by 10 years of dialysis, more than 90% of patients exhibit ACRD [9].

Patients with chronic renal failure on hemodialysis showed a significant presence of ACRD in our study. Approximately 19.9% of patients had ACRD. Recent studies described the strong relationship between ACRD, prolonged duration of dialysis, and renal cell carcinoma. [6]. In a comparative study, 148 patients (95 men and 53 women) underwent ultrasound assessment of the kidneys. ACRD was present in 20.3% of patients in that study (18.9% in men and 22.6% in women; p=.59) [10]. Although cystic renal disease is also found in general population with almost similar frequency. ACRD was also significantly common in patients receiving dialysis for three or more years than those with fewer than three years of dialysis (p=.001) [10].

In another longitudinal study, 30 patients on hemodialysis underwent serial CT scans of their abdomens. Seventeen patients (57%) had ACRD (mean dialysis length: 113.5 months), four patients (13%) had no renal cysts (mean dialysis length: 83.0 months), and nine patients (30%) had fewer than five renal cysts in each kidney (mean dialysis length, 21.5 months). Histologically confirmed RCC developed in two patients (7%) [11].

In another cross-sectional study, 37 patients with ESRD receiving hemodialysis underwent ultrasound (10 male patients, eight female patients, mean age of 50.4 years). Eighteen of the 37 patients (49%) had ACRD [12]. We found a similar frequency of ACRD in our study population.

The article "Frequency of Acquired Renal Cystic Disease in Patients on Long-Term Hemodialysis and Associated Renal Cell Carcinoma" was published in 2022. Journal: Cureus.

Most of the patients with ACRD (95%) had received more than three years of dialysis treatment, which supports findings from previous studies [10,12]. We also found that male patients were more affected than female patients, supporting findings from a previous study [13]. Another study found ACRD to be more common in patients older than age 60, which agrees with our findings [11]. ACRD was also more common in patients receiving dialysis twice per week, which matches a previous study [10]. Ninety percent of patients with kidneys smaller than 9 cm had ACRD, also reported in the literature [13].

Limitations

This was a cross-sectional study, and ultrasonography is not the gold standard for detecting cysts. Furthermore, we couldn't identify the link between ACRD and adequacy of dialysis, like measuring urea reduction ratio or Kt/V. But in limited-resource countries, ultrasound can be used as a screening tool. We were also limited by time constraints, as prolonging the study might have identified additional patients with ACRD or associated complications.

## Conclusions

Patient life expectancy for those with chronic renal failure is extending thanks to the availability of improved medical facilities and dialysis treatments. Long-term dialysis is associated with myriad complications ACRD is one of the complications of end-stage-renal disease irrespective of aetiopathogenesis. Since the frequency of ACRD increases with the duration of end-stage renal disease, so based on prior studies and our results, physicians should evaluate ACRD patients for RCC every year, especially if the patient has long-term disease duration treatment for over three years.
